# The DNA damage/repair cascade in glioblastoma cell lines after chemotherapeutic agent treatment

**DOI:** 10.3892/ijo.2015.2963

**Published:** 2015-04-16

**Authors:** LAURA ANNOVAZZI, VALENTINA CALDERA, MARTA MELLAI, CHIARA RIGANTI, LUIGI BATTAGLIA, DANIELA CHIRIO, ANTONIO MELCARNE, DAVIDE SCHIFFER

**Affiliations:** 1 Neuro-Bio-Oncology Center, Policlinico di Monza Foundation (Vercelli), I-13100 Vercelli, Italy; 2 Department of Oncology, University of Turin, I-10126 Turin, Italy; 3 Department of Drug Science and Technology, University of Turin, I-10125 Turin, Italy; 4 Department of Neurosurgery, CTO Hospital, Città della Salute e della Scienza, I-10126 Turin, Italy

**Keywords:** glioblastoma, glioma stem cells, DNA damage/repair, chemoresistance

## Abstract

Therapeutic resistance in glioblastoma multiforme (GBM) has been linked to a subpopulation of cells with stem cell-like properties, the glioma stem cells (GSCs), responsible for cancer progression and recurrence. This study investigated the *in vitro* cytotoxicity of three chemotherapeutics, temozolomide (TMZ), doxorubicin (Dox) and paclitaxel (PTX) on glioma cell lines, by analyzing the molecular mechanisms leading to DNA repair and cell resistance, or to cell death. The drugs were tested on 16 GBM cell lines, grown as neurospheres (NS) or adherent cells (AC), by studying DNA damage occurrence by Comet assay, the expression by immunofluorescence and western blotting of checkpoint/repair molecules and apoptosis. The three drugs were able to provoke a genotoxic injury and to inhibit dose- and time-dependently cell proliferation, more evidently in AC than in NS. The first cell response to DNA damage was the activation of the damage sensors (p-ATM, p-53BP1, γ-H2AX), followed by repair effectors; the expression of checkpoint/repair molecules appeared higher in NS than in AC. The non-homologous repair pathway (NHEJ) seemed more involved than the homologous one (HR). Apoptosis occurred after long treatment times, but only a small percentage of cells in NS underwent death, even at high drug concentration, whereas most cells survived in a quiescent state and resumed proliferation after drug removal. In tumor specimens, checkpoint/repair proteins were constitutively expressed in GBMs, but not in low-grade gliomas.

## Introduction

High-grade malignant gliomas are among the most rapidly growing and lethal human tumors. Despite multimodal therapies, the prognosis of glioblastoma multiforme (GBM) remains poor and the tumor inevitably recurs. The failure of therapeutic treatments is mainly due to the diffusion modalities of the tumor and to several resistance mechanisms of cancer cells, such as elevated expression of drug efflux transporters (1–3), reduced sensitivity to apoptotic signals and increased expression of growth factors. A pivotal role in resistance is played by the ability of tumor cells to repair DNA damage caused by radiation and chemotherapeutic agents, through a DNA damage response (DDR) cascade (4–8).

Multiple complex pathways occur in the eukaryotic cells for the surveillance and repair of genetic material and cell cycle control. To DNA damage the cancer cells respond with: i) cell cycle arrest and lesion repair; ii) entry into apoptosis or other cell deaths; iii) proliferation without repairing the damage favouring the effects of more genetic mutations. In response to genotoxic stress, cells do not progress through the cycle until the stability of the DNA molecule is ensured: the MRN (Mre11-Rad50-Nbs1) sensor complex recruits the protein kinases ataxia telangiectasia mutated (ATM) and ataxia telangiectasia Rad3-related (ATR), that initiate a transduction cascade activating downstream effectors, including H2AX histone, 53 binding protein 1 (53BP1) and the checkpoint kinases Checkpoint 1 (Chk1) and Checkpoint 2 (Chk2). These last two molecules act as a molecular switch determining, through phosphorylation of tumor suppressor protein p53, cell cycle arrest in order to allow DNA damage repair (Fig. 1A). If the damage is too extensive, apoptosis is triggered (9). Double strand breaks (DSBs), the most dangerous DNA lesions in mammalian cells, are repaired by two main pathways: homologous recombination (HR) and non-homologous end joining (NHEJ) (10,11). The former takes place only in actively cycling cells, during the S/G2 phases and its key effector is RAD51 protein. The latter occurs during G0/G1 phases and is driven by DNA-dependent protein kinase (DNA-PK), which consists of a regulatory subunit (Ku70/Ku80 heterodimer) and a catalytic subunit (DNA-PKcs) (Fig. 1A).

Glioma stem cells (GSCs), responsible for GBM growth and recurrence, show a relative resistance to apoptosis and an increased DNA repair capacity (12–14). Thanks to preferential activation of DDR and to an increased Chk1/Chk2 activity, a delayed cell cycle may be a major resistance mechanism (7) and Chk1/Chk2 inhibition is reported to sensitize to radio-treatments (13).

Temozolomide (TMZ), doxorubicin (Dox) and paclitaxel (PTX) are drugs commonly used in the clinical practice of solid tumors. TMZ, an alkylating agent at present employed in the standard therapy of GBM, induces methylation in multiple sites on DNA. The O^6^-methylguanines (O^6^-meGs) are the most cytotoxic adducts and are normally repaired by the O^6^-methylguanine-DNA methyltransferase (MGMT). The hypermethylation of the MGMT promoter determines epigenetic silencing of the protein and correlates with a better prognosis (15). If the cell is MGMT-deficient, a futile mismatch repair (MMR) cycle is triggered with formation of DNA DSBs and activation of ATM/ATR-Chk1/Chk2 signaling, G2/M-cell cycle arrest and ultimately apoptosis (16–18) (Fig. 1B). The anthracycline Dox interferes with cell growth by intercalation between DNA paired bases, finally causing cell death. PTX acts as antimitotic drug determining apoptosis. Also Dox and PTX are reported to induce DNA strand breaks and a repair response in some cell types (19,20); their use on brain tumors is limited due to the poor blood-brain barrier (BBB) penetration capacity, even though their *in vitro* effectiveness on GBM cells and in glioma animal models is proven (21–23).

The present study explored the *in vitro* effects of TMZ, Dox and PTX on primary GBM cell lines, focusing the attention on TMZ and by investigating DNA damage extent and the molecular mechanisms leading to a repair response, i.e., a resistant phenotype, or to cell death.

## Materials and methods

### Cell lines, culture conditions and tumor specimens

Primary human GBM cultures were established from tumors surgically resected at the Department of Neurosurgery of CTO Hospital (Turin, Italy). Malignant glioma U87-MG and 010627 cell lines were kindly supplied by Dr Rossella Galli (DIBIT San Raffaele, Milan, Italy). Ten cell lines were cultured, as previously described (24), in Dulbecco’s modified Eagle’s medium (DMEM)/F-12 supplemented with 20 ng/ml epidermal growth factor (EGF) and 10 ng/ml basic fibroblast growth factor (bFGF) for neurosphere (NS) assay and 6 cell lines in DMEM supplemented with 10% fetal bovine serum (FBS) for adherent cell (AC) growth (Table I). Both cultures were maintained at 37°C in 5% O_2_ and 5% CO_2_. All cell lines were characterized for MGMT gene promoter and p53 gene status (24,25) (Table I). Experiments with primary GBM lines were carried out using cells from passages 10–20 and cultures were checked for *Mycoplasma* contamination before use (e-Myco™ Mycoplasma PCR Detection kit, iNtRON Biotechnology, Korea). Formalin-fixed paraffin-embedded (FFPE) brain tumor samples were collected from 8 GBMs, one pilocytic astrocytoma and one oligodendroglioma. The histological diagnosis was performed according to World Health Organization (WHO) guidelines (26). The study was in compliance with the local institutional review board and Committee on Human Research and with the ethical human-subject standards of the World Medical Association Declaration of Helsinki Research. Written informed consent was obtained from all patients.

### Drug treatment and cytotoxicity assay

TMZ, Dox and PTX (all from Sigma-Aldrich Co., St. Louis, MO, USA) were dissolved in 100% dimethylsulfoxide (DMSO) for stock solutions. The final concentration of DMSO never exceeded 0.3% (v/v). All cell lines (10 NS and 6 AC) were treated with TMZ at increasing doses (5, 50, 100, 200 and 500 μM) and times [6, 24, 48, 72 and 120 hours (h)]; eleven cell lines (7 NS and 4 AC) were treated with 1, 2 and 5 μM Dox at 2, 24, 48 and 72 h; ten cell lines (7 NS and 3 AC) were treated with 10, 100, 1,000 and 5,000 nM PTX at 24, 48, 72 and 120 h. The drugs were added to dissociated NS cultures. After exposure, the cytotoxicity of the drugs was evaluated assessing the number of viable cells by the 3-(4,5-dimethylthiazol-2-yl)-2,5-diphenyl-tetrazolium bromide (MTT) assay (Roche, Diagnostic Corp., Indianapolis, IN, USA), measuring optical density at 570 nm (test wavelength) and 660 nm (reference wavelength) by a microplate spectrophotometer (Synergy HT, BioTek Instruments Inc., Winooski, VT, USA). For NS, cell counts were also performed by trypan blue using a TC20 automated cell counter (Bio-Rad, Berkeley, CA, USA). Cytotoxicity was expressed as number of surviving cells as percentage of control (untreated cells). The concentration of the drugs which caused a 50% inhibition of the cell growth, defined IC_50_, was calculated for each cell line at 72 h by non-linear regression from the survival curves of Fig. 2A.

### Comet assay

Cells were treated with different drug doses at various time-points and the occurrence of DNA damage induced by the drugs was investigated using the Comet (or single cell gel electrophoresis, SCGE) assay kit (Trevigen Inc., Gaithersburg, MD, USA) at neutral pH. Nuclei were labeled with SYBR Green I dye. Observations were made on a Zeiss Axioskop fluorescence microscope (Carl Zeiss, Oberkochen, Germany) equipped with an AxioCam5 MR5c and coupled to an Imaging system (AxioVision Release 4.5; Carl Zeiss). Cleaved DNA fragments caused by DSBs are detected as a tail (comet), the length of which is a measure of the DNA damage degree (27). Cells with comet tails were quantified as percentage over the total cell number and a visual score was assigned to the comets (28): score 0 representing undamaged cells (comets with no or barely detectable tails); score 1, 5–30% of migrated DNA; score 2, 31–70% of migrated DNA; score 3, >70% of migrated DNA (panel in Fig. 3G).

### Determination of apoptosis

Apoptosis was evaluated on cells after treatment with TMZ and PTX and on tissue sections by *in situ* terminal deoxynucleotidyl transferase-mediated dUTP-biotin nick end-labeling (TUNEL) assay, using the *in situ* cell death detection kit, fluorescein (Roche) according to the manufacturer’s protocols. Apoptotic indexes were calculated scoring 4 randomly selected fields and counting number of apoptotic cells over the total of viable cells which represented a quota in comparison with untreated cells.

### Immunofluorescence (IF)

IF was performed on NS and AC following TMZ and PTX treatments to monitor the activation of the damage/repair molecules p-ATM, p-Chk2, p-53BP1, γ-H2AX histone, HR effector RAD51, NHEJ effectors Ku70/Ku80 and DNA-PKcs. Cells were fixed for 20 min with 4% paraformaldehyde at room temperature, rinsed three times with PBS, blocked/permeabilized for 30 min with PBS containing 2% of the appropriate serum and 0.1% Triton X-100 and finally stained with the following primary antibodies: monoclonal mouse anti-human γ-H2AX (Ser139) (05-636; Millipore, Bedford, MA, USA; dilution 1:200), monoclonal mouse anti-human p-ATM (Ser1981) (05-740; Millipore; dilution 1:100), polyclonal rabbit anti-human p-Chk2 (Thr68) (BK2197S; Cell Signaling Technology, Beverly, MA, USA; dilution 1:100), polyclonal rabbit anti-human p-53BP1 (Ser25) (IHC-00053; Bethyl Laboratories, Inc., Montgomery, TX, USA; dilution 1:200), monoclonal mouse anti-human RAD51 (MS-988; NeoMarkers, Fremont, CA, USA; dilution 1:100), monoclonal mouse anti-human DNA-PKcs (MS-423; NeoMarkers; dilution 1:100) and monoclonal mouse anti-human Ku70/Ku80 (MS-286; NeoMarkers; dilution 1:200). Negative controls were obtained by omitting the primary antibody. Alexa Fluor^®^ 488-AffiniPure goat anti-rabbit IgG and Alexa Fluor^®^ 594-AffiniPure rabbit anti-mouse IgG (Jackson ImmunoResearch Laboratories, Inc., West Grove, PA, USA) were used as secondary antibodies. Cell nuclei were stained with 4′,6-diamidino-2-phenylindole (DAPI) and examined under a Zeiss Axioskop fluorescence microscope.

### Immunocytochemistry (ICC) and ımmunohistochemistry (IHC)

Due to the interfering spontaneous fluorescence of Dox, ICC, instead of IF, was carried out on cells treated with Dox. IHC was performed on the 8 GBM and 2 low-grade tissues. The analyses were made using a Ventana Full BenchMark^®^ XT automated immunostainer (Ventana Medical Systems Inc., Tucson, AZ, USA) and UltraView™ Universal DAB Detection kit (Ventana Medical Systems Inc.) as detection system. Heat-induced epitope retrieval (HIER) was performed in Tris-EDTA, pH 8.0. Primary antibodies were the same used for IF with the same dilutions. Negative controls were obtained by omitting the primary antibody.

### Western blotting (WB)

WB was performed as previously described (24) using the following primary antibodies: monoclonal mouse anti-human γ-H2AX (Ser139) (05-636; Millipore; dilution 1:1,000), monoclonal mouse anti-human p-ATM (Ser1981) (05-740; Millipore; dilution 1:2,000), polyclonal rabbit anti-human p-Chk2 (Thr68) (BK2197S; Cell Signaling Technology; dilution 1:1,000), monoclonal mouse anti-human RAD51 (MS-988; NeoMarkers; dilution 1:500), and monoclonal mouse anti-human Ku70/Ku80 (MS-286; NeoMarkers; dilution 1:1,000). A polyclonal rabbit anti-human α-tubulin (LF-PA0146; LabFrontier, Seoul, Korea; dilution 1:5,000) was used to normalize sample loading and transfer.

### Statistical analysis

The level of significance was determined by a two-tailed Student’s t-test. All quantitative data presented are the average value ± standard error (SE) from at least three independent determinations. Statistical significance was defined as p<0.05 or p<0.01.

## Results

### Cytotoxicity studies on GBM cell lines after TMZ, Dox and PTX treatments

NS lines were self-renewing, clonogenic, multipotent and expressing undifferentiation antigens; AC displayed a differentiation antigen profile (24). TMZ, Dox and PTX inhibited cell proliferation, both in NS and in AC by MTT assay, controlled by trypan blue method. The cytotoxic effect of the three drugs were dose- and time-dependent and more evident on AC than on NS (Fig. 2A-a-f). NS were resistant to dosages of TMZ <10 μM, with the exception of CV10 and CV21 lines, that presented hypermethylation of MGMT promoter (Table I). Even high TMZ concentrations resulted in the survival of ≤30% of the cells in some NS lines. On the contrary, on most AC, TMZ concentrations <50 μM reduced cell growth to 50% after 72-h exposure. Compared with growth of untreated NS and AC (Fig. 2B-a and -f, respectively, from NO3 cell line, taken as a representative line), cell proliferation in NS (Fig. 2B-b-e) and AC adhesion (Fig. 2B-g-j) was hindered by TMZ in a dose and time-dependent manner. However, the growth inhibition in NS was not irreversible and the depletion of cells was not complete, even at high drug dosages. Even after 5-day treatment with high TMZ dosage (200 μM), a few single cells survived re-acquiring growth capacity within one month after treatment suspension (Fig. 2B-k and -l).

Dox uptake by NS and AC was evident in most cells already after 2 h with 2 μM drug and, after 24-h exposure, the number of viable cells showed 20% decrease with inhibition of clonogenicity in NS and of cell adhesion in AC. After 72-h treatment, 80% cells were dead. Also 100 nM PTX at 48 h inhibited evidently cell proliferation both in NS and in AC. After 5-day treatment a few single cells of NS lines survived re-acquiring growth capacity within one month after treatment suspension.

### Evaluation of DNA damage by Comet assay

By Comet assay no damage was detectable on untreated NS (Fig. 3A) and AC (data not shown) and on NS treated with 50 μM TMZ for 24 h (Fig. 3B); a comet tail was evident only after 72-h exposure with 50 μM drug (Fig. 3C): >10% of cells showed a score-2-length tail. Comets with score-3 length were visible in >50% of cells treated with 200 μM TMZ (Fig. 3D). The damage resulted more elevated in AC and in NS lines with methylated MGMT promoter. DNA lesions were revealed in NS (Fig. 3E) and even more in AC (data not shown) with 2 μM Dox at 72 h and the same effect but weaker was observed after 72-h treatment with 100 nM PTX both in NS (Fig. 3F) and in AC (data not shown) with score-2 length tails. Quantification of cell damage by Comet assay in untreated and treated NO3 NS is reported in Fig. 3G.

### Determination of cell apoptosis induced by drug treatment

Apoptosis was a late phenomenon, evident only after 72-h drug exposure, both in NS and AC (Fig. 4A and B). The frequency of apoptotic cells following treatment with increasing concentrations of TMZ for 6, 24 and 72 h is shown in Fig. 4C and D for NS and AC, respectively. In treated NS, apoptosis did not exceed 10–15% and it was ≤30% in AC. PTX-induced apoptosis was evidenced at 72 h already at concentration of 10 nM. At the highest drug dosages, the percentage of apoptotic cells was ≤20% in NS (Fig. 4E) and ≤30% in AC (Fig. 4F).

### Studies of checkpoint/repair pathways in treated cells

The antigens of repair cascade resulted negative in untreated NS, with the exception of p-ATM, γ-H2AX, Ku70/Ku80, DNA-PKcs, moderately expressed in some lines (Fig. 5A-a-g). No expression was shown in untreated AC (Fig. 5B-a-g). The expression of all the sensors and effectors, except RAD51, was evident after 48-h exposure to 100 μM TMZ, both in NS and, at a minor extent, in AC (Fig. 5A and B-h-n). Expression of p-ATM, γ-H2AX, p-Chk2, Ku70/80 and RAD51 in 4 NS lines treated with TMZ was confirmed by WB analysis (Fig. 5D). Dox effects were the same as TMZ but earlier. γ-H2AX, indicator of DSBs, was evident after 48-h treatment with 50 μM TMZ or 5 μM Dox, both in NS and in AC. Concurrent administration of the two drugs increased the effect with γ-H2AX expressed in ~90% of cells and a significant decrease in cell number (Fig. 5E-a-d for NS and -e-h for AC). All repair markers became negative after 72 h with high drug concentrations (500 μM TMZ or 5 μM Dox): cells were dying or no longer able to activate the repair cascade. After 72-h treatment with 100 nM PTX, a moderate activation of checkpoint/repair response with a mild expression of all markers except RAD51 was found in NS, whereas, interestingly, in treated AC, several cells appeared arrested in metaphase and with a strong expression of p-ATM, p-Chk2, p-53BP1, γ-H2AX, DNA-PKcs, Ku70/Ku80 (Fig. 5C-a-g). After 24 h from the beginning of treatments, the presence of activated damage sensors (p-ATM, p-53BP1, γ-H2AX, p-Chk2) was more evident, whereas at longer times (72 h), expression level of effectors (DNA-PKcs, Ku70/80) increased and that of sensor molecules decreased as repair proceeded (Fig. 5F).

### Studies of checkpoint/repair and apoptosis in glioma tissues

p-ATM, γ-H2AX and the key proteins of NHEJ system, DNA-PKcs and Ku70/Ku80, were constitutively expressed in the GBM specimens studied, particularly in proliferation areas and in perinecrotic pseudopalisades (Fig. 6A-a, -b, -e and -f). p-ATM and γ-H2AX were sometimes positive in macrophages and reactive astrocytes. p-Chk2 and RAD51 expression was rather scarce and heterogeneous (Fig. 6A-c and -d) and p-53BP1 was not detectable. The two low-grade glioma tissues analyzed were almost negative for the markers, with the exception of p-ATM and γ-H2AX, poorly positive at level of mitoses (Fig. 6B). Apoptosis occurred in the palisades of circumscribed necroses and was scattered in the proliferating areas of GBM (29) (Fig. 6C).

## Discussion

In this study we demonstrated that three commonly used anticancer drugs, TMZ, Dox and PTX, were able, under *in vitro* conditions, to reduce significantly the number of viable cells in GBM NS lines and even more in AC lines, inhibiting clonogenic growth in the former and hindering cell adhesion in the latter. The finding, as for TMZ, is in agreement with recent reports (30,31). Dox and PTX caused a more evident reduction of cell viability in comparison with TMZ, both in NS and in AC. IC_50_ values for TMZ and Dox at 72 h were, on average, higher for NS than for AC, proving that the former are more resistant than the latter, characterized by a more differentiated state. No significant differences in IC_50_ values for PTX was observed between NS and AC.

Cell lines with a hypermethylated MGMT promoter were mostly more sensitive to TMZ, but the data were in some cases discordant. MGMT expression indeed is not the only factor to be considered in evaluating TMZ response: p53 wild-type status is reported as fundamental to determine cell cycle arrest and the entry in the apoptotic process (32,33). In our data, among the cell lines with hypermethylated MGMT those with mutated p53 gene appeared more resistant to the action of TMZ than the ones with wild-type p53.

In NS cultures treated with TMZ or PTX, the depletion of cells was never complete even at high drug dosages; cells could resist the drugs in a non-proliferating state, as already observed for TMZ (30,31) and resumed proliferation within 1–2 months after treatment suspension. The maintenance of a quiescent state and metabolic inertia may, therefore, represent a mechanism of genome protection in GSCs; the consequence is that antineoplastic treatments can have a cytostatic rather than a cytotoxic effect. Dox effect was more lethal and irreversible.

Apoptosis following treatments was a late phenomenon demonstrable only after 72 h, as already reported (18,34). In our observations, it was more evident in AC than in NS, but in both cases the frequency of apoptosis does not explain the level of reduction of viable cells, in agreement with the data of Beier *et al* (35).

By Comet assay we found that TMZ, Dox and, to lesser extent, PTX were able to produce in glioma cells a DNA damage, that increased proportionally with drug doses and times and was higher in AC than in NS lines, with the consequent activation of the checkpoint/repair pathways. Moreover, we noted in some untreated NS lines a basal expression of some checkpoint/repair proteins, which was significantly elicited following drug exposure. After DNA injury also AC were able to trigger a repair response, although to a minor extent. Sensors of damage were the first proteins to be activated and they decreased with time, as the effectors increased and repair of lesions took place. From our data, NHEJ repair system activity seemed higher than the one of HR. It was reported that high tumor levels of DNA-PK correlate with poor survival in GBM patients treated with postsurgical radiation (36).

In GBM tissue specimens, we found a constitutive expression of checkpoint/repair proteins, not present in the low-grade tumors. At the beginning of tumorigenesis, DDR machinery acts as a protective mechanism against glioma progression, limiting the expansion of malignant clones with unstable genome (37). In glioma pathogenesis an aberrant constitutive activation of repair mechanisms was reported in response to DNA replication stress produced by oncogenes (38).

In conclusion, cell fate after treatments depends on the preferential activation of repair or apoptotic pathways. The intrinsic resistance to genotoxic therapies of malignant glioma cells could therefore be explained on one hand, by their ability to stop growth and survive in a quiescent state and, on the other hand, by the involvement of an enhanced DNA damage signaling. Moreover, we demonstrated that also Dox and PTX would be effective cytotoxic/cytostatic agents, similarly to TMZ, on glioma cells and, once the way to cross the BBB is found (39,40), they could be potentially useful in the GBM treatment. Targeted inhibition of the DNA repair factors could, therefore, be useful to sensitize malignant gliomas to genotoxic treatments and to improve therapeutic strategies.

## Figures and Tables

**Figure 1:** Scheme of cell checkpoint/repair signaling after DNA damage (A) and mechanisms of cytotoxicity of TMZ (B) [modified from Bolderson *et al* (10) and Sarkaria *et al* (8)].

**Figure 2:** Cytotoxic effect of TMZ, Dox and PTX on glioma cells. (A) Cell viability in neurospheres (NS) and adherent cells (AC) calculated at 72 h after the addition of various doses of TMZ (a and b), Dox (c and d) and PTX (e and f). Data are mean values ± SE of three independent experiments, each performed in triplicate. (B) Inhibitory effect of TMZ increasing doses (5, 50, 100 and 200 μM) at 72 h on NO3 NS (b-e) and on NO3 AC (g-j) growth; untreated NS and AC in (a) and (f), respectively; few surviving cells of NO3 NS line after 120-h treatment with 200 μM TMZ (k) and proliferation restarting after 30 days from treatment suspension (l). All ×100 magnification.

**Figure 3:** Comet assay on NO3 NS line. Comet assay on: untreated NO3 NS (A); NS after 50 μM TMZ for 24 h (B); after 50 μM TMZ for 72 h (C); after 200 μM TMZ for 72 h (D); after 2 μM Dox for 72 h (E); after 100 nM PTX for 72 h (F). Quantification of DNA damage in untreated cells (control) of NO3 NS and after 72-h treatment with TMZ, Dox and PTX at various doses (G), by using an arbitrary visual score (upper panel); data are mean values ± SE of three independent experiments, each performed in triplicate.

**Figure 4:** Evaluation of apoptosis in treated cells. Apoptosis after 100 μM TMZ for 72 h in NO3 NS (A) and in NO3 AC (B); TUNEL labeling, nuclei counterstained with DAPI, ×400. Quantification of apoptotic cells after treatment with different doses and times of TMZ in NO3 NS (C) and AC (D) and after treatment with different doses and times of PTX in NO3 NS (E) and AC (F). Data are mean values ± SE of three independent experiments, each performed in triplicate. ^*,**^Statistical significance (p<0.05 and p<0.01, two-tailed Student’s t-test).

**Figure 5:** Study of checkpoint/repair response in NO3 NS and AC. (A) Expression by immunofluorescence of checkpoint/repair proteins in untreated NO3 NS (a-g) and in cells treated with 100 μM TMZ for 48 h (h-n). (B) The same as above in untreated (a-g) and treated NO3 AC (h-n). (C) The same as above in NO3 AC treated with 100 nM PTX for 72 h (a-g): positivity of the antigens is evident at metaphasis level. Nuclei counterstained with DAPI. All ×200 magnification. (D) Expression by western blotting of p-ATM, p-Chk2, γ-H2AX and Ku70/Ku80 in 4 NS lines (CV10, 010627, CV21 and NO3), untreated and treated with 100 μM TMZ for 48 h. No band for RAD51 was detectable in any lines, not even after TMZ treatment. (E) Expression by immunocytochemistry of γ-H2AX, as indicator of DNA damage, in untreated NO3 NS (a, ×400) and AC (e, ×400) and after 50 μM TMZ for 48 h [(b) and (f) for NS and AC, respectively, ×400], after 5 μM Dox for 48 h [(c) and (g) for NS and AC, respectively, ×400] and after combined treatment with 50 μM TMZ and 5 μM Dox for 48 h [(d) and (h) for NS and AC, ×400 and ×630, respectively]. (F) Levels of checkpoint/repair proteins at 24 (a) and 72 h (b) in NO3 NS, untreated (control) and treated with 100 μM TMZ, 2 μM Dox or 100 nM PTX.

**Figure 6:** (A) Immunohistochemical expression in GBM tissues of p-ATM, DAB, ×200 (a); γ-H2AX, DAB, ×200 (b); p-Chk2, DAB, ×400 (c); RAD51, positive in scattered cells, DAB, ×400 (d); DNA-PKcs, DAB, ×200 (e); Ku70/Ku80, DAB, ×200 (f). (B) Immunohistochemical expression of p-ATM in a pilocytic astrocytoma, DAB, ×400 (a); γ-H2AX in an oligodendroglioma, DAB, ×200 (b); p-Chk2 in an oligodendroglioma, DAB, ×400 (c); RAD51 in an oligodendroglioma, DAB, ×400 (d); DNA-PKcs in an oligodendroglioma, DAB, ×200 (e); Ku70/Ku80 in an oligodendroglioma, DAB, ×200 (f). (C) Evaluation of apoptosis in GBM tissue sections. Scattered apoptotic nuclei in palisades of circumscribed necroses (a) and in proliferating areas (b) of a GBM sample, TUNEL labeling, ×400.

**Table I:** Cell lines with the IC_50_ values for each drug and the MGMT and p53 gene status.

Cell line	IC_50_ (μM)^a^ for TMZ	IC_50_ (μM)^a^ for Dox	IC_50_ (μM)^a^ for PTX	Methylation status of MGMT promoter	Status of p53 gene
U87-MG NS	170	0.92	-	Methylated	Wild-type
010627 NS	135	-	-	Methylated	Mutated
CV10 NS	8.5	-	-	Methylated	Wild-type
CV21 NS	44	0.68	0.03	Methylated	Wild-type
NO3 NS	120	0.85	0.044	Unmethylated	Wild-type
NO4 NS	100	0.98	0.1	Methylated	Mutated
NO6 NS	170	-	0.0094	Unmethylated	Wild-type
CTO3 NS	97	1.85	0.066	Methylated	Mutated
CTO5 NS	130	1.18	0.08	Unmethylated	Wild-type
CTO15 NS	130	0.65	0.035	Unmethylated	Mutated
U87-MG AC	42	0.72	-	Methylated	Wild-type
010627 AC	130	-	-	Methylated	Mutated
CV10 AC	5	-	-	Methylated	Wild-type
NO3 AC	72	0.78	0.05	Unmethylated	Wild-type
CTO3 AC	50	0.83	0.077	Methylated	Mutated
CTO15 AC	46	0.67	0.027	Unmethylated	Mutated

a IC_50_ was calculated at 72 h.

## References

[1] Caldera V, Mellai M, Annovazzi L, Monzeglio O, Piazzi A, Schiffer D (2012). MGMT hypermethylation and MDR system in glioblastoma cancer stem cells. Cancer Genomics Proteomics.

[2] Salmaggi A, Boiardi A, Gelati M, Russo A, Calatozzolo C, Ciusani E, Sciacca FL, Ottolina A, Parati EA, La Porta C, Alessandri G, Marras C, Croci D, De Rossi M (2006). Glioblastoma-derived tumorospheres identify a population of tumor stem-like cells with angiogenic potential and enhanced multidrug resistance phenotype. Glia.

[3] Johannessen TC, Bjerkvig R (2012). Molecular mechanisms of temozolomide resistance in glioblastoma multiforme. Expert Rev Anticancer Ther.

[4] Alexander BM, Pinnell N, Wen PY, D’Andrea A (2012). Targeting DNA repair and the cell cycle in glioblastoma. J Neurooncol.

[5] Schmalz PG, Shen MJ, Park JK (2011). Treatment resistance mechanisms of malignant glioma tumor stem cells. Cancers (Basel).

[6] Frosina G (2010). The bright and the dark sides of DNA repair in stem cells. J Biomed Biotechnol.

[7] Frosina G (2009). DNA repair and resistance of gliomas to chemotherapy and radiotherapy. Mol Cancer Res.

[8] Sarkaria JN, Kitange GJ, James CD, Plummer R, Calvert H, Weller M, Wick W (2008). Mechanisms of chemoresistance to alkylating agents in malignant glioma. Clin Cancer Res.

[9] Kastan MB, Bartek J (2004). Cell-cycle checkpoints and cancer. Nature.

[10] Bolderson E, Richard DJ, Zhou BB, Khanna KK (2009). Recent advances in cancer therapy targeting proteins involved in DNA double-strand break repair. Clin Cancer Res.

[11] Pardo B, Gómez-González B, Aguilera A (2009). DNA repair in mammalian cells: DNA double-strand break repair: how to fix a broken relationship. Cell Mol Life Sci.

[12] Johannessen TC, Bjerkvig R, Tysnes BB (2008). DNA repair and cancer stem-like cells--potential partners in glioma drug resistance?. Cancer Treat Rev.

[13] Bao S, Wu Q, McLendon RE, Hao Y, Shi Q, Hjelmeland AB, Dewhirst MW, Bigner DD, Rich JN (2006). Glioma stem cells promote radioresistance by preferential activation of the DNA damage response. Nature.

[14] Liu G, Yuan X, Zeng Z, Tunici P, Ng H, Abdulkadir IR, Lu L, Irvin D, Black KL, Yu JS (2006). Analysis of gene expression and chemoresistance of CD133^+^ cancer stem cells in glioblastoma. Mol Cancer.

[15] Hegi ME, Diserens AC, Gorlia T, Hamou MF, de Tribolet N, Weller M, Kros JM, Hainfellner JA, Mason W, Mariani L (2005). MGMT gene silencing and benefit from temozolomide in glioblastoma. N Engl J Med.

[16] Hirose Y, Berger MS, Pieper RO (2001). p53 effects both the duration of G2/M arrest and the fate of temozolomide-treated human glioblastoma cells. Cancer Res.

[17] Günther W, Pawlak E, Damasceno R, Arnold H, Terzis AJ (2003). Temozolomide induces apoptosis and senescence in glioma cells cultured as multicellular spheroids. Br J Cancer.

[18] Roos WP, Batista LF, Naumann SC, Wick W, Weller M, Menck CF, Kaina B (2007). Apoptosis in malignant glioma cells triggered by the temozolomide-induced DNA lesion O6-methylguanine. Oncogene.

[19] Kurz EU, Douglas P, Lees-Miller SP (2004). Doxorubicin activates ATM-dependent phosphorylation of multiple downstream targets in part through the generation of reactive oxygen species. J Biol Chem.

[20] Branham MT, Nadin SB, Vargas-Roig LM, Ciocca DR (2004). DNA damage induced by paclitaxel and DNA repair capability of peripheral blood lymphocytes as evaluated by the alkaline comet assay. Mutat Res.

[21] Stan AC, Casares S, Radu D, Walter GF, Brumeanu TD (1999). Doxorubicin-induced cell death in highly invasive human gliomas. Anticancer Res.

[22] Lesniak MS, Upadhyay U, Goodwin R, Tyler B, Brem H (2005). Local delivery of doxorubicin for the treatment of malignant brain tumors in rats. Anticancer Res.

[23] Chang SM, Kuhn JG, Robins HI, Schold SC, Spence AM, Berger MS, Mehta M, Pollack IF, Rankin C, Prados MD (2001). A Phase II study of paclitaxel in patients with recurrent malignant glioma using different doses depending upon the concomitant use of anticonvulsants: A North American Brain Tumor Consortium report. Cancer.

[24] Caldera V, Mellai M, Annovazzi L, Piazzi A, Lanotte M, Cassoni P, Schiffer D (2011). Antigenic and genotypic similarity between primary glioblastomas and their derived neurospheres. J Oncol.

[25] Mellai M, Monzeglio O, Piazzi A, Caldera V, Annovazzi L, Cassoni P, Valente G, Cordera S, Mocellini C, Schiffer D (2012). MGMT promoter hypermethylation and its associations with genetic alterations in a series of 350 brain tumors. J Neurooncol.

[26] Louis DN, Ohgaki H, Wiestler OD, Cavanee WK (2007). WHO Classification of Tumors of the Central Nervous Systems.

[27] Singh NP, McCoy MT, Tice RR, Schneider EL (1988). A simple technique for quantitation of low levels of DNA damage in individual cells. Exp Cell Res.

[28] Collins AR, Oscoz AA, Brunborg G, Gaivão I, Giovannelli L, Kruszewski M, Smith CC, Stetina R (2008). The comet assay: Topical issues. Mutagenesis.

[29] Mellai M, Schiffer D (2007). Apoptosis in brain tumors: Prognostic and therapeutic considerations. Anticancer Res.

[30] Beier D, Röhrl S, Pillai DR, Schwarz S, Kunz-Schughart LA, Leukel P, Proescholdt M, Brawanski A, Bogdahn U, Trampe-Kieslich A (2008). Temozolomide preferentially depletes cancer stem cells in glioblastoma. Cancer Res.

[31] Mihaliak AM, Gilbert CA, Li L, Daou MC, Moser RP, Reeves A, Cochran BH, Ross AH (2010). Clinically relevant doses of chemotherapy agents reversibly block formation of glioblastoma neurospheres. Cancer Lett.

[32] Hermisson M, Klumpp A, Wick W, Wischhusen J, Nagel G, Roos W, Kaina B, Weller M (2006). O6-methylguanine DNA methyltransferase and p53 status predict temozolomide sensitivity in human malignant glioma cells. J Neurochem.

[33] Bocangel DB, Finkelstein S, Schold SC, Bhakat KK, Mitra S, Kokkinakis DM (2002). Multifaceted resistance of gliomas to temozolomide. Clin Cancer Res.

[34] Knizhnik AV, Roos WP, Nikolova T, Quiros S, Tomaszowski KH, Christmann M, Kaina B (2013). Survival and death strategies in glioma cells: Autophagy, senescence and apoptosis triggered by a single type of temozolomide-induced DNA damage. PLoS One.

[35] Beier D, Schriefer B, Brawanski K, Hau P, Weis J, Schulz JB, Beier CP (2012). Efficacy of clinically relevant temozolomide dosing schemes in glioblastoma cancer stem cell lines. J Neurooncol.

[36] Kase M, Vardja M, Lipping A, Asser T, Jaal J (2011). Impact of PARP-1 and DNA-PK expression on survival in patients with glioblastoma multiforme. Radiother Oncol.

[37] Bartek J, Bartkova J, Lukas J (2007). DNA damage signalling guards against activated oncogenes and tumour progression. Oncogene.

[38] Bartkova J, Hamerlik P, Stockhausen MT, Ehrmann J, Hlobilkova A, Laursen H, Kalita O, Kolar Z, Poulsen HS, Broholm H (2010). Replication stress and oxidative damage contribute to aberrant constitutive activation of DNA damage signalling in human gliomas. Oncogene.

[39] Battaglia L, Gallarate M, Peira E, Chirio D, Muntoni E, Biasibetti E, Capucchio MT, Valazza A, Panciani PP, Lanotte M (2014). Solid lipid nanoparticles for potential doxorubicin delivery in glioblastoma treatment: Preliminary in vitro studies. J Pharm Sci.

[40] Chirio D, Gallarate M, Peira E, Battaglia L, Muntoni E, Riganti C, Biasibetti E, Capucchio MT, Valazza A, Panciani P (2014). Positive-charged solid lipid nanoparticles as paclitaxel drug delivery system in glioblastoma treatment. Eur J Pharm Biopharm.

